RETRACTED

# Establishment and Validation for Predicting the Death of Multiple Myeloma among Whites

**DOI:** 10.1155/2022/3050199

**Published:** 2022-08-16

**Authors:** Jian Tao, Ling Wang, Liyu Zhang, Zheyun Gu, Xiaodan Zhou

**Affiliations:** Department of Hematology, The Second Affiliated Hospital of Nantong University, Nantong 226001, Jiangsu, China

## Abstract

The prognosis of multiple myeloma (MM) patients was poor in white-American patients as compared to black-American patients. This study aimed to predict the death of MM patients in whites based on the National Cancer Institute's Surveillance, Epidemiology, and End Results (SEER) database. A total of 28,912 white MM patients were included in this study. Data were randomly divided into a training set and a test set (7 : 3). The random forest and 5-fold cross-validation were used for developing a prediction model. The performance of the model was determined by calculating the area under the curve (AUC) with 95% confidence interval (CI). MM patients in the death group had older age, higher proportion of tumor distant metastasis, bone marrow as the disease site, receiving radiotherapy, and lower proportion of receiving chemotherapy than that in the survival group (all *P* < 0.001). The AUC of the random forest model in the training set and testing set was 0.741 (95% CI, 0.740–0.741) and 0.703 (95% CI, 0.703–0.704), respectively. In addition, the AUC of the age-based model was 0.688 (95% CI, 0.688–0.689) in the testing set. The results of the DeLong test indicated that the random forest model had better predictive effect than the age-based model (*Z* = 7.023, *P* < 0.001). Further validation was performed based on age and marital status. The results presented that the random forest model was robust in different age and marital status. The random forest model had a good performance to predict the death risk of MM patients in whites.

## 1. Introduction

Multiple myeloma (MM) is a plasma cell dyscrasia and accounts for 10% of all hematological malignancies [1, 2]. The global age-standardized incidence rate of MM was 2.1 per 100,000 people in 2016 [3]. In the US, the age-standardized incidence rate of MM during the same period was higher than that in the global rate with 7.1 per 100,000 people [4], and incidence rate is gradually increasing [5]. In 2021, 34,920 new cases of MM were diagnosed, and approximately 15,600 patients died from the disease [6]. MM has caused a significant burden of disease worldwide [3]. Therefore, accurately predicting the death risk of MM patients can help physicians to intervene in advance to improve the prognosis of patients.

Many factors including age, gender, family history, radiation exposure, racial, and biomarkers have an important impact on the incidence and prognosis of patients with MM [7–10]. Previous studies found that the prognosis and prevalence of MM patients are different between white-Americans and black-Americans [11,12]. Waxman et al. indicated that white-Americans with MM had a poorer survival as compared to black-Americans [13]. However, the risk of death in white MM patients has not received widespread attention. Establishing a prognostic tool in white patients with MM may help clinicians identify patients at risk of death in advance and intervene early to improve patient survival. Perrot et al. used a prognostic index based on six cytogenetic markers to identify the risk of death in patients with MM [14]. Zhou et al. used long noncoding RNA signatures of four biomarkers to predict overall survival in patients with MM [15]. However, these prognostic tools for overall MM patients were based on complex biological markers or small sample sizes [14–16]. In clinical practice, a simple and applicable prediction tool for predicting the death risk of MM patients based on large sample size is needed.

RETRACTED

Herein, this study aimed to develop a model to predict the death of MM patients in whites. This prediction model was established based on the National Cancer Institute's Surveillance, Epidemiology, and End Results (SEER) database with a large sample size.

## 2. Methods

### 2.1. Study Design and Population

All data were extracted from the original 18 registries of the SEER database (https://seer.cancer.gov/), which contains data from 18 geographically diverse populations representing rural, urban, and regional populations. SEER 18 database includes approximately 27.8% of the US population. Cases were diagnosed from 2007 to 2016, and MM was defined by the International Classification of Diseases for Oncology, Third Edition (ICD-O-3) (histology code: 9731, 9732, 9734) [17]. Inclusion criteria were as follows: (1) age ≥18 years; (2) whites; (3) patients who were diagnosed with MM. Excluded criteria were as follows: (1) various types of tumors; (2) nonprimary MM; (3) patients with incomplete data. Because the data used in this study were accessed from the SEER 18 database (a publicly available database), the Institutional Review Board of The First People's Hospital of Nantong was not required.

### 2.2. Data Collection

Demographic and clinical data of MM patients were collected from the SEER database including age, gender (male and female), marital status (married, single, widowed, and others), number of malignant tumors in situ, number of benign tumors (=0 and >0), metastasis (distant and others), disease site (bone marrow and others), chemotherapy (yes or no), radiotherapy (yes or no), and survival state (alive and dead). The death of patients was the outcome indicator. Patients were divided into the survival group and death group according to their survival status at the end of follow-up.

RETRACTED

### 2.3. Statistical Analysis

All statistical analyses were the two-side test, and *P* < 0.05 was considered statistical difference. The software SAS 9.4 (SAS Institute Inc., Cary, NC, USA) and Python 3.8 (Python Software Foundation, Delaware, USA) was used for statistical analysis. Continuous variables with normal distribution were expressed as mean ± standard deviation (SD), and the *t*-test was used for comparison between groups; nonnormal variables were expressed as a median and interquartile range (M (Q1, Q3)), the Mann–Whitney U rank-sum test was used for comparison between groups. Categorical variables were expressed as numbers and percentages (*n* (%)), and the Chi-square test (*χ*^2^) or the Fisher's test was used for comparison between groups.

The random forest was used to develop a prediction model. All data were randomly divided into the training set, and the test is set with a ratio of 7 : 3. The training set data were used for model development, and the test set data were used for internal validation. The method of randomization was performed using SAS 9.4 software. According to the number of patients included in the study, serial numbers were generated after setting random seeds in SAS. The first 70% of the serial numbers were divided into the training set, and the last 30% were divided into the test set. The 5-fold cross-validation was performed, which is currently a common technique in data mining. The model performance was quantified by calculating the area under the curve (AUC) with 95% confidence interval (CI), as well as accuracy, sensitivity, specificity, positive predictive value (PPV), and negative predictive value (NPV). The selection of the optimal was based on the AUC value of the model, and the parameter corresponding to the maximum AUC value is the optimal model parameter. The parameter range of the random forest model was the number of decision trees (500) and the depth of decision tree (10).

## 3. Results

### 3.1. Baseline Characteristics of Study Population

A total of 28,912 white patients with MM were included in this study (Figure 1). Of these patients, 20,238 (70%) were divided into the training set, with mean age of 67.28 ± 12.05 years and 11,598 (57.31%) cases were males. Among these patients in the training set, 12,878 (63.63%) were married, 2,420 (11.96%) were single, and 2,950 (14.58%) were widowed. The mean number of malignant tumors in situ was 1.08 ± 0.30, and the median overall survival was 28.00 (11.00, 55.00) months. In total, the disease site of 19,001 (93.89%) patients was bone marrow, 19,155 (94.65%) had distant metastases, 12,183 (60.20%) patients received chemotherapy, and 15,826 (78.20%) received radiotherapy. At the end of the follow-up, 9,437 (46.63%) patients were alive, and 10,801 (53.37%) patients died. Detailed characteristics of the study population are shown in Table 1.

RETRACTED

### 3.2. Comparison of Differences between the Training Set and Test Set

A total of 28,912 white patients were randomly divided into the training set and the test set with a ratio of 7 : 3. The difference analysis showed that no statistical difference was observed in all characteristics between the training set data and the test set data (Supplement Table 1). These results indicated that the data of the training set and the test set were balanced, and the data of the test set can be used to test the model of the training set.

### 3.3. Comparison of Characteristics between the Survival Group and the Death Group

Univariate analysis showed that age (*t* = −50.310, *P* < 0.001), the proportion of tumor distant metastasis (*χ*^2^ = 172.869, *P* < 0.001), bone marrow as the disease site (*χ*^2^ = 149.955, *P* < 0.001), and receiving radiotherapy (*χ*^2^ = 16.682, *P* < 0.001) were higher in the death group than in the survival group. Compared with the survival group, the proportion of receiving chemotherapy was lower in the death group (*χ*^2^ = 63.150, *P* < 0.001). There was a statistical difference in marital status (*χ*^2^ = 632.686, *P* < 0.001) between the two groups (Table 2).

### 3.4. Establishment and Validation of the Model

The random forest was used to develop the prediction model. The important variables for the random forest model were age, marital status, metastasis, disease site, etc.; especially, age was the most important variable in the random forest model (Figure 2).

The performances of the all-variable model and age-based model in the training set and testing set are displayed in Table 3. The AUC of the all-variable model in the training set and the testing set was 0.741 (95% CI, 0.740–0.741) and 0.703 (95% CI, 0.703–0.704), respectively. The accuracy and specificity of the all-variable model in the testing set were 0.641 (95% CI, 0.631–0.651) and 0.700 (95% CI, 0.686–0.714), respectively. Furthermore, the AUC of the age-based model in the training set and testing set was 0.697 (95% CI, 0.697–0.698) and 0.688 (95% CI, 0.688–0.689), respectively. The results of the DeLong test indicated that the random forest model had a better predictive effect than the age-based model (*Z* = 7.023, *P* < 0.001). The ROC curves and calibration curve of the model in the training set and testing set are presented in Figures 3 and 4.

RETRACTED

### 3.5. Further Validation Based on Age and Marital Status

Age and marital status were important variables for the random forest model, and further validation was performed based on age and marital status.  Table 4 demonstrates the performance of the random forest models in age and marital status subgroups. The AUC of the model in patients aged ≥65 years, <65 years, single, widowed, married, and others marital status was 0.681 (95% CI, 0.681–0.682), 0.614 (95% CI, 0.613–0.614), 0.662 (95% CI, 0.661–0.663), 0.693 (95% CI, 0.693–0.693), 0.642 (95% CI, 0.641–0.644), and 0.695 (95% CI, 0.694–0.696), respectively. The prediction effect of the random forest model was robust in different ages and marital statuses.

## 4. Discussion

In this study, a random forest model was established to predict the death risk of MM patients among whites. The important variables of the model were age, marital status, metastasis, disease site, etc., and age was the most important variable in the model. The AUC of the random forest model in the training set and test set were 0.741 and 0.703, respectively. This indicated that our random forest model had good predictive ability for death risk in white MM patients, and the model was robust. The AUC of the age-based model was 0.688, suggesting that age may be an important predictor of death risk in white patients with MM. The results of the DeLong test indicated that the random forest model had better predictive effect than the age-based model. Further validation showed that the prediction effect of the random forest model was robust in different age and marital status.

The prognosis of MM is widely heterogeneous, patients survive for more than 10 years after diagnosis, while others died within a few months [14]. Furthermore, the incidence and prognosis of MM have race differences. It was reported that the incidence rates of MM among black-American patients are about twice that of white-American patients [18, 19], but black-American patients with MM had better survival as compared to white-American patients [13]. This study developed a random forest model to predict the death of MM among whites. The AUC of the model in the training set and test set were 0.741 and 0.703, respectively, indicating the model had good performance in predicting the death of MM patients among whites. Hájek et al. conducted a novel risk stratification algorithm to estimate the risk of death in patients with relapsed MM patients, and the C-index of their model was 0.715 [20]. The study of Terebelo et al. established a prediction matrix to predict the early mortality of MM patients [16]. Perrot et al. developed a prognostic model of newly diagnosed MM patients based on six cytogenetic abnormalities, and their results showed that a higher prognostic index was consistently associated with a poor survival outcome [14]. However, few studies have predicted the death of MM patients in whites. Our study provided a random forest model to predict the death risk of MM patients among whites, which may help clinicians make early interventions to improve the prognosis of patients.

RETRACTED

In our model, age played the most important role in predicting the death of MM patients among whites. The AUC of the single variable age model was 0.688 in our study. Aging is related to the reduction of reparative and regenerative potential in tissues and organs [21, 22]. These changes affect the pharmacokinetics and pharmacodynamics of drugs, increase toxicity, and reduce clinical efficacy and treatment tolerance [23]. It was reported that the incidence of MM is higher in older patients, with 63% of patients aged 65 years and over, and only 0.02–0.3% of patients under 30 years [24]. The study of Augustson et al. indicated that 60% of MM patients who died within 2 months of starting treatment were over 65 years [25]. In further validation, 65 years was chosen as the threshold, and the random forest model was performed to predict the death of MM patients among different age populations. The results found that the prediction effect of the model was better for the population ≥65 years than of the population <65 years, but the prediction effects of these two models were not as good as the model of the overall population model.

Our results indicated that marital status also was associated with the death of MM patients. An extensive analysis of more common cancers based on the SEER database showed that unmarried patients, including those who are widowed, are more likely to suffer from metastatic cancer, undertreatment, and death from cancer than married patients [26]. The study of Costa et al. found that, among MM patients, being single, widowed, or divorced led to a higher risk of death [27]. A possible explanation is that, after being diagnosed with cancer, married patients displayed less distress, depression, and anxiety than unmarried patients because their partners can share emotions and provide social support [28]. In clinical practice, special attention should be paid to widowed, divorced, or single MM patients and beware of death.

To the best of our knowledge, this study was the first to predict the death risk of MM patients in whites. We established a random forest model using simple clinical characteristics of MM patients. This model may help clinicians predict the death of MM patients in whites and make early interventions to improve the prognosis of patients. However, this study has some limitations. First, this prediction model was developed based on the US SEER database and may not be suitable for all whites. Second, the internal validation results showed that the model fit well, but external validation of the prediction models was necessary when it was used in clinical practice. Third, some clinical biochemical indicators such as serum creatinine and *β*2-microglobulin may be associated with the prognosis of patients with MM [29, 30], but these biochemical indicators were not included in our model due to the lack of these data in the database.

RETRACTED

## 5. Conclusions

A random forest model was established to predict the death of MM patients in whites based on the SEER database. Age and marital status were the important variables for predicting the death of MM patients in whites. Further validation indicated that the prediction effect of the random forest model was robust in different age and marital status. Our model may provide a tool to predict the death risk of MM patients in whites, which may help clinicians with early intervention to improve patient outcomes.

## Figures and Tables

**Figure 1:** The flow chart of patients screening. All white patients with MM included in the study were randomly divided into a training set and a test set in a ratio of 7 : 3 for the model establishment and validation, respectively.

**Figure 2:** Variable importance of random forest model for predicting the risk of death in white multiple myeloma (MM) patients. The variable importance of random forests indicates which variables contributed the most to the final model.

**Figure 3:** Performance and evaluation of random forest model in the training set. (a) Receiver operator characteristic (ROC) curves; (b) calibration curves.

**Figure 4:** Performance and evaluation of random forest model in the testing set. (a) Receiver operator characteristic (ROC) curves; (b) calibration curves.

**Table 1:** Characteristics of included patients in the training set.

Variables	Total (*n* = 20238)
Age, years, mean ± SD	67.28 ± 12.05

*Gender, n (%)*	
Female	8640 (42.69)
Male	11598 (57.31)

*Marital status, n (%)*	
Married	12878 (63.63)
Single	2420 (11.96)
Widowed	2950 (14.58)
Others	1990 (9.83)

Number of malignant tumors in situ, mean ± SD	1.08 ± 0.30
*Number of benign tumors, n (%)*	
0	20131 (99.47)
>0	107 (0.53)

*Metastasis, n (%)*	
Distant	19155 (94.65)
Others	1083 (5.35)

*Disease site, n (%)*	
Bone marrow	19001 (93.89)
Others	1237 (6.11)

*Chemotherapy, n (%)*	
No	8055 (39.80)
Yes	12183 (60.20)

*Radiotherapy, n (%)*	
No	4412 (21.80)
Yes	15826 (78.20)

*Survival state, n (%)*	
Alive	9437 (46.63)
Dead	10801 (53.37)
Overall survival, months, M (Q1, Q3)	28.00 (11.00, 55.00)

RETRACTED

**Table 2:** Univariate analysis between the survival group and the death group in the training set.

Variables	Total (*n* = 20238)	Survival group (*n* = 9437)	Death group (*n* = 10801)	Statistic	*P*
Age, years, mean ± SD	67.28 ± 12.05	62.97 ± 11.52	71.04 ± 11.21	*t* = -50.310	<0.001

Gender, *n* (%)				*χ* ^2^ = 0.101	0.751
Female	8640 (42.69)	4040 (42.81)	4600 (42.59)		
Male	11598 (57.31)	5397 (57.19)	6201 (57.41)		

Marital status, *n* (%)				*χ* ^2^ = 632.686	<0.001
Married	12878 (63.63)	6595 (69.88)	6283 (58.17)		
Single	2420 (11.96)	1182 (12.53)	1238 (11.46)		
Widowed	2950 (14.58)	759 (8.04)	2191 (20.29)		
Others	1990 (9.83)	901 (9.55)	1089 (10.08)		

Number of malignant tumors in situ, mean ± SD	1.08 ± 0.30	1.08 ± 0.30	1.08 ± 0.30	*t* = 0.460	0.643

Number of benign tumors, *n* (%)				*χ* ^2^ = 0.316	0.574
0	20131 (99.47)	9390 (99.50)	10741 (99.44)		
>0	107 (0.53)	47 (0.50)	60 (0.56)		

Metastasis, *n* (%)				*χ* ^2^ = 172.869	<0.001
Distant	19155 (94.65)	8722 (92.42)	10433 (96.59)		
Others	1083 (5.35)	715 (7.58)	368 (3.41)		

Disease site, *n* (%)				*χ* ^2^ = 149.955	<0.001
Bone marrow	19001 (93.89)	8652 (91.68)	10349 (95.82)		
Others	1237 (6.11)	785 (8.32)	452 (4.18)		

Chemotherapy, *n* (%)				*χ* ^2^ = 63.150	<0.001
No	8055 (39.80)	3480 (36.88)	4575 (42.36)		
Yes	12183 (60.20)	5957 (63.12)	6226 (57.64)		

Radiotherapy, *n* (%)				*χ* ^2^ = 16.682	<0.001
No	4412 (21.80)	2177 (23.07)	2235 (20.69)		
Yes	15826 (78.20)	7260 (76.93)	8566 (79.31)		

**Table 3:** The performance of the random forest model.

Group	Parameter (95% CI)	All-variable model	Age-based model
*Training set*			
	AUC	0.741 (0.740–0.741)	0.697 (0.697–0.698)
	Accuracy	0.673 (0.667–0.680)	0.641 (0.635–0.648)
	Sensitivity	0.612 (0.603–0.621)	0.533 (0.523–0.542)
	Specificity	0.744 (0.735–0.752)	0.765 (0.757–0.774)
	PPV	0.732 (0.723–0.741)	0.722 (0.712–0.732)
	NPV	0.626 (0.617–0.635)	0.589 (0.580–0.597)

*Testing set*			
	AUC	0.703 (0.703–0.704)	0.688 (0.688–0.689)
	Accuracy	0.641 (0.631–0.651)	0.636 (0.626–0.646)
	Sensitivity	0.591 (0.576–0.605)	0.533 (0.518–0.547)
	Specificity	0.700 (0.686–0.714)	0.754 (0.741–0.768)
	PPV	0.694 (0.680–0.708)	0.714 (0.699–0.729)
	NPV	0.597 (0.583–0.611)	0.583 (0.570–0.597)

Note: CI: confidence interval; AUC: area under the curve; PPV: positive predictive value; NPV: negative predictive value.

**Table 4:** The performance of the random forest models in age and marital status subgroups.

Subgroup	Parameter (95% CI)	All-variable models
*Age ≥65 years*		
	AUC	0.681(0.681–0.682)
	Accuracy	0.647(0.634–0.660)
	Sensitivity	0.725(0.710–0.741)
	Specificity	0.511(0.489–0.533)
	PPV	0.721(0.705–0.736)
	NPV	0.517(0.495–0.540)

*Age <65 years*		
	AUC	0.614(0.613–0.614)
	Accuracy	0.621(0.604–0.637)
	Sensitivity	0.030(0.021–0.039)
	Specificity	0.986(0.981–0.991)
	PPV	0.565(0.448–0.682)
	NPV	0.622(0.605–0.638)

*Single marital status*		
	AUC	0.662(0.661–0.663)
	Accuracy	0.583(0.553–0.613)
	Sensitivity	0.367(0.326–0.408)
	Specificity	0.817(0.783–0.851)
	PPV	0.684(0.630–0.738)
	NPV	0.544(0.508–0.580)

*Widowed marital status*		
	AUC	0.693(0.693–0.693)
	Accuracy	0.636(0.623–0.648)
	Sensitivity	0.461(0.442–0.480)
	Specificity	0.807(0.793–0.822)
	PPV	0.701(0.680–0.723)
	NPV	0.604(0.588–0.620)

*Others marital status*		
	AUC	0.695(0.694–0.696)
	Accuracy	0.724(0.699–0.748)
	Sensitivity	0.886(0.865–0.907)
	Specificity	0.305(0.257–0.353)
	PPV	0.767(0.741–0.792)
	NPV	0.509(0.442–0.577)

*Married marital status*		
	AUC	0.642(0.641–0.644)
	Accuracy	0.583(0.550–0.615)
	Sensitivity	0.433(0.389–0.477)
	Specificity	0.756(0.715–0.797)
	PPV	0.673(0.621–0.725)
	NPV	0.535(0.494–0.575)

RETRACTED

## Data Availability

Data used and analyzed in this study are available from SEER database (https://seer.cancer.gov/).

## Supplementary Materials

Supplementary Materials Supplement Table 1: comparison between the training set and testing set.
